The article "Applying Dynamic Systems to Social Media by Using Controlling Stability" was retracted in 2023. Reasons: unreliable results or conclusions; concerns about the data; concerns about the results or conclusions; concerns about the peer review.

# Applying Dynamic Systems to Social Media by Using Controlling Stability

**DOI:** 10.1155/2022/4569879

**Published:** 2022-01-31

**Authors:** Abdulsattar Abdullah Hamad, M. Lellis Thivagar, Malik Bader Alazzam, Fawaz Alassery, Fahima Hajjej, Ali A. Shihab

**Affiliations:** ^1^School of Mathematics Madurai Kamaraj University, Madurai, India; ^2^Faculty of Computer Science and Informatics, Amman Arab University, Amman, Jordan; ^3^Department of Computer Engineering, College of Computers and Information Technology, Taif University, P.O. Box 11099, Taif 21944, Saudi Arabia; ^4^Department of Information Systems, College of Computer and Information Sciences, Princess Nourah bint Abdulrahman University, P.O. Box 84428, Riyadh 11671, Saudi Arabia; ^5^Mathematics Department, Education for Pure Sciences College, Tikrit University, Tikrit, Iraq

## Abstract

This study focuses on hybrid synchronization, a new synchronization phenomenon in which one element of the system is synced with another part of the system that is not allowing full synchronization and nonsynchronization to coexist in the system. When $\underset{t⟶\infty }{\lim}Y-\alpha X=0$, where *Y* and *X* are the state vectors of the drive and response systems, respectively, and Wan (*α* = ∓1)), the two systems' hybrid synchronization phenomena are realized mathematically. Nonlinear control is used to create four alternative error stabilization controllers that are based on two basic tools: Lyapunov stability theory and the linearization approach.

## 1. Introduction

Alazzam et al.' study [1] is an example. Control and hybrid three-dimensional synchronization (HPS) procedures are for a unique hyperchaotic system. To begin, the revolutionary hyperchaotic system is regulated to an unstable equilibrium position or limit cycle using only one scalar controller with two state variables. Using Lyapunov's direct approach, the HPS between two new hyperchaotic systems is studied. A nonlinear feedback vector controller is presented to establish perfect synchronization between two new hyperchaotic systems, which can then be condensed further into a single scalar controller. Finally, simulation data are supplied to ensure the effectiveness of these strategies.

The proposed approaches have some implications for lowering controller installation costs and complexity. Dynamical systems have received a lot of attention. It is one of the first attempts in a Lu model, and a new hyperchaotic model with three unstable equilibrium points is disclosed. Despite the fact that the newly built system is basic, it is six-dimensional (6D) and has eighteen terms in 2021. [2]. It presents the new structure of high dimension (6D), novel king of quaternion complete, and has some unusual properties [3–6]. There is another study which introduces another chaotic and hyperchaotic complex nonlinear, and this type has a significant stake in its phase-space behavior [7–9]. It has been organized in the previous time, for example, a 3D auto system, which is not differ-isomorphic with the Lorenz attractor. In the arrangement of values for a parameter *k*, [10] has proposed another 3D attractor that shows chaotic behavior in distinct respects and not diffeomorphic with Lorenz [11–18]. The first chaotic nonlinear system has been suggested by Lorenz [19–22] in which is a generalization of the Lorenz system. The Lorenz system's messy structure is utilized.

The article "Applying Dynamic Systems to Social Media by Using Controlling Stability" was retracted in 2023. Reasons: unreliable results or conclusions; concerns about the data; concerns about the results or conclusions; concerns about the peer review.

## 2. Hybrid Synchronization between Two Similar Systems

We have already learned about the dynamic system [18], which is in the following formula:

(1) $$\begin{array}{c} \left\{\begin{array}{c} \;{\dot{x}}_{1}=a\left(x_{2}-x_{1}\right)+x_{4},\\ {\dot{x}}_{2}=cx_{1}-x_{2}-x_{1}x_{3}+x_{5},\\ {\dot{x}}_{3}=-bx_{3}+x_{1}x_{2},\\ {\dot{x}}_{4}=dx_{4}-x_{1}x_{3},\\ {\dot{x}}_{5}=-kx_{2},\\ {\dot{x}}_{6}=hx_{6}+rx_{2}, \end{array}\right. \end{array}$$

which represents the driving system as *x*_1_,  *x*_2_,  *x*_3_,  *x*_4_, *x*_5_,  *x*_6_ are the variables representing the system states and that *a*, *b*, *c*, *d*, *k*, *h*, and *r* are the real positive parameters and their values are 11, 7/3, 27, 2, 7.4, 1, and 1, respectively.

While, the response system can be written as follows:

(2) $$\begin{array}{c} \left\{\begin{array}{c} {\dot{y}}_{1}=a\left(y_{2}-y_{1}\right)+y_{4}+u_{1},\\ {\dot{y}}_{2}=cy_{1}-y_{2}-y_{1}y_{3}+y_{5}+u_{2},\\ {\dot{y}}_{3}=-by_{3}+y_{1}y_{2}+u_{3},\\ {\dot{y}}_{4}=dy_{4}-y_{1}y_{3}+u_{4},\\ {\dot{y}}_{5}=-ky_{2}+u_{5},\\ {\dot{y}}_{6}=hy_{6}+ry_{2}+u_{6}. \end{array}\right. \end{array}$$

The dynamic error of the hybrid synchronization between the 6D chaos system (1) and system (2) is defined by the following relationship.

(3) $$\begin{array}{c} e_{i}=y_{i}-x_{i},\;i=1,3,5⟶\underset{t⟶\infty }{\lim}e_{i}=0,\\ e_{j}=y_{j}+x_{j},\;j=2,4,6⟶\underset{t⟶\infty }{\lim}e_{j}=0. \end{array}$$

Thus, the error is calculated for the dynamic system as follows:

(4) $$\begin{array}{c} \left\{\begin{array}{c} {\dot{e}}_{1}=ae_{2}-ae_{1}+e_{4}-2ax_{2}-2x_{4}+u_{1},\\ {\dot{e}}_{2}=ce_{1}-e_{2}+e_{5}-y_{1}e_{3}+x_{3}e_{1}-2y_{1}x_{3}+2cx_{1}+2x_{5}+u_{2},\\ {\dot{e}}_{3}=-be_{3}+e_{1}e_{2}-x_{2}e_{1}+x_{1}e_{2}-2x_{1}x_{2}+u_{3},\\ {\dot{e}}_{4}=de_{4}-y_{1}e_{3}+x_{3}e_{1}-2y_{1}x_{3}+u_{4},\\ {\dot{e}}_{5}=-ke_{2}+2kx_{2}+u_{5},\\ {\dot{e}}_{6}=he_{6}+re_{2}+u_{6}. \end{array}\right. \end{array}$$

Using the method of linear approximation to find the characteristic equation and the intrinsic values of the system before the control, which is witnessing a state of instability for the system before the control, this method confirms this thing.

(5) $$\begin{array}{c} \lambda^{6}+\frac{31}{3}\lambda^{5}-\frac{3069}{15}\lambda^{4}+\frac{1558}{15}\lambda^{3}+\frac{64004}{15}\lambda^{2}-\frac{8496}{5}\lambda -348=0,\\ \left\{\begin{array}{c} \lambda_{1}=2,\;\\ \lambda_{2}=1,\\ \lambda_{3}=-\frac{7}{3},\;\\ \lambda_{4}=10.9659-8.10^{-9}i,\\ \lambda_{5}=\;-12.6916-3.92820323010^{-9}i,\\ \lambda_{6}=\;0.3257+8.92820323010^{-9}i. \end{array}\right. \end{array}$$

The results of the distinctive equation confirm that the error of the dynamic system is in the position of instability.

The article "Applying Dynamic Systems to Social Media by Using Controlling Stability" was retracted in 2023. Reasons: unreliable results or conclusions; concerns about the data; concerns about the results or conclusions; concerns about the peer review.

**Theorem 1 .**

Let *U* be the controller of the system:

(6) $$\begin{array}{c} \left\{\begin{array}{c} u_{1}=2ax_{2}+2x_{4}-ce_{2}-x_{3}e_{2}+x_{2}e_{3}-x_{3}e_{4},\\ u_{2}=-ae_{1}+\;2y_{1}x_{3}-2cx_{1}-2x_{5}-x_{1}e_{3}+ke_{5}-re_{6},\\ u_{3}=y_{1}e_{2}-e_{1}e_{2}+2x_{1}x_{2}+y_{1}e_{4},\\ u_{4}=-2\;de_{4}-e_{1}+2y_{1}x_{3},\\ u_{5}=-e_{2}-2kx_{2}-e_{5},\\ u_{6}=-2he_{6}. \end{array}\right. \end{array}$$

Thus, the hybrid synchronization between system (1) and system (2) can be observed in two ways:

**Proof**

After compensating the control (6) in the dynamic system error (4), we get

(7) $$\begin{array}{c} \left\{\begin{array}{c} {\dot{e}}_{1}=ae_{2}-ae_{1}+e_{4}-ce_{2}-x_{3}e_{2}+x_{2}e_{3}-x_{3}e_{4},\\ {\dot{e}}_{2}=ce_{1}-e_{2}+e_{5}-y_{1}e_{3}+x_{3}e_{1}-ae_{1}-x_{1}e_{3}+ke_{5}-re_{6},\\ {\dot{e}}_{3}=-be_{3}-x_{2}e_{1}+x_{1}e_{2}+y_{1}e_{2}+y_{1}e_{4},\\ {\dot{e}}_{4}=-de_{4}-y_{1}e_{3}+x_{3}e_{1}-e_{1},\\ {\dot{e}}_{5}=-ke_{2}-e_{2}-e_{5},\\ {\dot{e}}_{6}=re_{2}-he_{6}. \end{array}\right. \end{array}$$

The first method is the method of linear approximation:

(8) $$\begin{array}{c} \lambda^{6}+\frac{53}{3}\lambda^{5}+\frac{12834}{25}\lambda^{4}+\frac{286498}{75}\lambda^{3}+\frac{286609}{25}\lambda^{2}+\frac{373231}{25}\lambda +\frac{169704}{25}=0,\\ \left\{\begin{array}{c} \lambda_{1}=-1,\\ \lambda_{2}=-\frac{7}{3},\\ \lambda_{3}=-2.3511,\\ \lambda_{4}=-2.6530,\\ \lambda_{5}=-\;4.4979+\;19.6945\;i,\\ \lambda_{6}=-\;4.4979-\;19.6945\;i. \end{array}\right. \end{array}$$

The linear approximation method succeeded in systems 1 and 2 showing the hybrid synchronization between the two systems and the Lyapunov Method is failed. We get $\dot{V}\left(e_{i}\right)$ as follows:

And they use the Lebanov method [18–20], as follows.

After differentiating the function *V*(*e*_*i*_), we get

(9) $$\begin{array}{c} \dot{V}\left(e\right)=e_{1}\left(\;ae_{2}-ae_{1}+e_{4}-\text{c}e_{2}-x_{3}e_{2}+x_{2}e_{3}-x_{3}e_{4}\right)\\ +e_{2}\left(ce_{1}-e_{2}+e_{5}-\;y_{1}e_{3}+x_{3}e_{1}-ae_{1}-x_{1}e_{3}+ke_{5}-re_{6}\right)\\ +e_{3}\left(-be_{3}-x_{2}e_{1}+x_{1}e_{2}+\;y_{1}e_{2}+y_{1}e_{4}\right)+e_{4}\left(-de_{4}-y_{1}e_{3}+x_{3}e_{1}-e_{1}\right)\\ +e_{5}\left(-ke_{2}-e_{2}-e_{5}\right)+\;e_{6}\left(re_{2}-he_{6}\right),\\ \dot{V}\left(e_{i}\right)=-ae_{1}^{2}-e_{2}^{2}-be_{3}^{2}-de_{4}^{2}-e_{5}^{2}-he_{6}^{2}=-e_{i}^{T}\;Q_{0_{4}}e_{i},\\ Q_{0_{4}}=\;diag\left(a,1,b,d,1,h\right). \end{array}$$

Thus, **Q**_0_4__ > 0, and this leads to $\dot{V}\left(e_{i}\right)$ being negatively defined in **R**^6^. Thus, the nonlinear control unit is suitable, in which there is no synchronization.

The article "Applying Dynamic Systems to Social Media by Using Controlling Stability" was retracted in 2023. Reasons: unreliable results or conclusions; concerns about the data; concerns about the results or conclusions; concerns about the peer review.

The initial values (2, 1, 8, 6, 12, 4), (−18, −9, −1, −5, −20, 15) are used to illustrate how the hybrid synchronization occurs between the two systems (1) and (2). Figures 1 and 2 and (2) show the verification of these results numerically.

**Theorem 2 .**

The nonlinear U control of system (4) and Figure 3 is designed as follows:

(10) $$\begin{array}{c} \left\{\begin{array}{c} u_{1}=2ax_{2}+2x_{4}-ce_{2}-x_{3}e_{2}+x_{2}e_{3}-x_{3}e_{4},\\ u_{2}=-ae_{1}+2y_{1}x_{3}-2cx_{1}-2x_{5}-x_{1}e_{3}-e_{6},\\ u_{3}=y_{1}e_{2}-e_{1}e_{2}+2x_{1}x_{2}+y_{1}e_{4},\\ u_{4}=-2\;de_{4}-e_{1}+2y_{1}x_{3},\\ u_{5}=-2kx_{2}-e_{5},\\ u_{6}=-2he_{6}. \end{array}\right. \end{array}$$

The hybrid synchronization between the two systems (1) and (2) can be explained in two ways.

**Proof**

By relying on control (10) with system (4),

(11) $$\begin{array}{c} \left\{\begin{array}{c} {\dot{e}}_{1}=ae_{2}-ae_{1}+e_{4}-ce_{2}-x_{3}e_{2}+x_{2}e_{3}-x_{3}e_{4},\\ {\dot{e}}_{2}=ce_{1}-e_{2}+e_{5}-y_{1}e_{3}+x_{3}e_{1}-ae_{1}-x_{1}e_{3}-e_{6},\\ {\dot{e}}_{3}=-be_{3}-x_{2}e_{1}+x_{1}e_{2}+y_{1}e_{2}+y_{1}e_{4},\\ {\dot{e}}_{4}=-de_{4}-y_{1}e_{3}+x_{3}e_{1}-e_{1},\\ {\dot{e}}_{5}=-ke_{2}-e_{5},\\ {\dot{e}}_{6}=-he_{6}+re_{2}. \end{array}\right. \end{array}$$

The first method is the method of linear approximation:

(12) $$\begin{array}{c} \lambda^{6}+\frac{53}{3}\lambda^{5}+\frac{2167}{5}\lambda^{4}+\frac{38509}{15}\lambda^{3}+\frac{90806}{15}\lambda^{2}+\frac{31068}{5}\lambda +\frac{11552}{5}=0,\\ \left\{\begin{array}{c} \lambda_{1}=-1,\\ \lambda_{2}=-\frac{7}{3},\\ \lambda_{3}=-1.2965,\\ \lambda_{4}=-1.9544,\\ \lambda_{5}=-\;5.3745+\;17.6928i,\\ \lambda_{6}=-\;5.3745-\;17.6928i. \end{array}\right) \end{array}$$

The linear approximation method succeeded in showing the hybrid synchronization between the two systems.

The second method is the method of Lebanov.

The Lebanov derivative with control (10) is as follows:

(13) $$\begin{array}{c} \dot{V}\left(e\right)=-ae_{1}^{2}-e_{2}^{2}-be_{3}^{2}-de_{4}^{2}-e_{5}^{2}-he_{6}^{2}+e_{2}e_{5}\left(1-k\right)+e_{2}e_{6}\left(r-1\right)=-e^{T}Q_{1}\;e. \end{array}$$

So, we get the matrix

(14) $$\begin{array}{c} Q_{1_{4}}=\left[\begin{array}{cccccc} a & 0 & 0 & 0 & 0 & 0\\ 0 & 1 & 0 & 0 & \left(\frac{\left(k-1\right)}{2}\right) & \frac{\left(1-r\right)}{2}\\ 0 & 0 & b & 0 & 0 & 0\\ 0 & 0 & 0 & d & 0 & 0\\ 0 & \frac{\left(k-1\right)}{2} & 0 & 0 & 1 & 0\\ 0 & \frac{\left(1-r\right)}{2} & 0 & 0 & 0 & h \end{array}\right]. \end{array}$$

The matrix *Q*_1_4__) is nondiagonal.

The article "Applying Dynamic Systems to Social Media by Using Controlling Stability" was retracted in 2023. Reasons: unreliable results or conclusions; concerns about the data; concerns about the results or conclusions; concerns about the peer review.

Now, find the parameters to confirm that the array is negatively defined.

(15) $$\begin{array}{c} \left\{\begin{array}{cc} 1, & a>0,\\ 2, & b>0,\\ 3, & d>0,\\ 4, & 1>\frac{{\left(k-1\right)}^{2}}{4},\\ 5, & \;\left(h-\frac{h{\left(k-1\right)}^{2}}{4}-\frac{{\left(1-r\right)}^{2}}{4}\right)>0. \end{array}\right. \end{array}$$

There are some inequalities that are not correct, and therefore, *Q*_1_4__ is negatively defined, so the control failed to achieve hybrid synchronization between the two systems, and to overcome this problem, we update the P-matrix with the same control as follows:

(16) $$\begin{array}{c} \;P_{1_{4}}=diag\left(\frac{1}{2},\frac{1}{2},\frac{1}{2},\frac{1}{2},\frac{5}{84},\frac{1}{2}\right). \end{array}$$

The simulation was implemented via the wolf algorithm and MATLAB software 2020, with parameters *a*=11, *b*=−7/3, *c*=25, *d*=2, *h*=9.1, *r*=1, *p*=1, *q*=2 and control parameter *k*=13.5, and the new model has five +ve Lyapunov spectra.

The derivative of Lebanov is as follows:

(17) $$\begin{array}{c} \;\dot{V}\left(e_{i}\right)=-10e_{1}^{2}-e_{2}^{2}-\frac{8}{3}e_{3}^{2}-2e_{4}^{2}-\frac{5}{42}e_{5}^{2}-e_{6}^{2}=\;-e^{T}Q_{2_{4}}e, \end{array}$$

such that *Q*_2_4__=*di*  *ag*(10,1, 8/3, 2, 5/42, 1); it is a positive definition matrix, thus achieving hybrid synchronization between the two systems (1) and (2) [23] Figure 4 shows the numerical validity of what we have arrived at results.

## 3. Conclusion

In Figure 2, the convergence system of the complete synchronization scheme, we focused on the nonlinear control strategy, and another method was suggested, namely, linearization; in addition, we used the Lyapunov method which is adopted in all previous works in order to compare and verify between the two methods.

The results show that the linearization method is the best for achieving the synchronization since the stability Lyapunov method needs to construct an auxiliary function (Lyapunov function) and may need to update this function sometimes. At other times, it is difficult for us to create a suitable auxiliary function which leads to the fall of this method; thus, the failure and success of the method depend on the additional auxiliary factor, in addition to the control factor. While, the linearization method dispenses for this auxiliary factor, which gives it extra strength compression of the stability of the Lyapunov method. It also addressed the issue of known parameters and unknown.

The article "Applying Dynamic Systems to Social Media by Using Controlling Stability" was retracted in 2023. Reasons: unreliable results or conclusions; concerns about the data; concerns about the results or conclusions; concerns about the peer review.

As for the phenomenon of projective synchronization, which is the most comprehensive among the phenomena, we were only using the method of Lyapunov in achieving the phenomenon, and the results were good.

## Figures and Tables

**Figure 1:** Hybrid synchronization between two systems (1).

**Figure 2:** The convergence of system (4) with control (10).

**Figure 3:** The convergence of system (4).

**Figure 4:** Hybrid synchronization between the two systems (1).

## Data Availability

The data used to support the findings of this study are included within the article.
